# Proteomic analysis of the rice (*Oryza officinalis*) provides clues on molecular tagging of proteins for brown planthopper resistance

**DOI:** 10.1186/s12870-018-1622-9

**Published:** 2019-01-18

**Authors:** Xiaoyun Zhang, Fuyou Yin, Suqin Xiao, Chunmiao Jiang, Tengqiong Yu, Ling Chen, Xue Ke, Qiaofang Zhong, Zaiquan Cheng, Weijiao Li

**Affiliations:** 1 Yunnan Provincial Key Lab of Agricultural Biotechnology, Key Lab of Southwestern Crop Gene Resources and Germplasm Innovation, Ministry of Agriculture, Kunming, Yunnan People’s Republic of China; 2 Biotechnology and Germplasm Resources Institute, Yunnan Academy of Agricultural Sciences, Kunming, Yunnan People’s Republic of China; 3 Faculty of Chinese Materia Medica, Yunnan University of Traditional Chinese Medicine, Kunming, Yunnan People’s Republic of China

**Keywords:** Rice, Brown planthopper (BPH), Proteomics, Resistance, Molecular mechanism

## Abstract

**Background:**

Among various pests, the brown planthopper (BPH) that damages rice is the major destructive pests. Understanding resistance mechanisms is a critical step toward effective control of BPH. This study investigates the proteomics of BPH interactions with three rice cultivars: the first resistant (PR) to BPH, the second susceptible (PS), and the third hybrid (HR) between the two, in order to understand mechanisms of BPH resistance in rice.

**Results:**

Over 4900 proteins were identified from these three rice cultivars using iTRAQ proteomics study. A total of 414, 425 and 470 differentially expressed proteins (DEPs) were detected from PR, PS and HR, respectively, after BPH infestation. Identified DEPs are mainly enriched in categories related with biosynthesis of secondary metabolites, carbon metabolism, and glyoxylate and dicarboxylate metabolism. A two-component response regulator protein (ORR22) may participate in the early signal transduction after BPH infestation. In the case of the resistant rice cultivar (PR), 6 DEPs, i.e. two lipoxygenases (LOXs), a lipase, two dirigent proteins (DIRs) and an Ent-cassa-12,15-diene synthase (OsDTC1) are related to inheritable BPH resistance. A heat shock protein (HSP20) may take part in the physiological response to BPH infestation, making it a potential target for marker-assisted selection (MAS) of rice. Quantitative real-time polymerase chain reaction (qRT-PCR) revealed eight genes encoding various metabolic proteins involved in BPH resistance. During grain development the expressions of these genes varied at the transcriptional and translational levels.

**Conclusions:**

This study provides comprehensive details of key proteins under compatible and incompatible interactions during BPH infestation, which will be useful for further investigation of the molecular basis of rice resistance to BPH and for breeding BPH-resistant rice cultivars.

**Electronic supplementary material:**

The online version of this article (10.1186/s12870-018-1622-9) contains supplementary material, which is available to authorized users.

## Background

For over 3.5 billion people rice has been a major food, supplying > 20% of the dietary calorie intake for humans across the globe. The Asia–Pacific region, mainly China, India, Indonesia, and Vietnam produces over 90% of the rice available to the world [1]. In these areas, the brown planthopper (BPH) *Nilaparvata lugens* (Stål) (Hemiptera: Delphacidae) turn to be the major insect pest destructiong the produce. BPH is a herbivore pest that attacks only on rice plants (monophagous) and usually feeds on vascular sap. It sucks the phloem sap from leaf sheath of rice plants using a stylet, leading to hopper burn and in most severe cases kills the entire plant during flowering [2]. BPH can also transmit plant viruses causing additional damage to rice plants [3]. BPH has caused devastating damages to rice crops in recent years. In China alone, 1–1.5 billion kg of rice production is lost annually due to BPH infestation, equivalent to a loss of several billion Yuans (CNY) in economic terms [4]. The extensive use of chemical insecticides has become the most common method for the control of BPH, which has resulted in many problems, including toxicity to its natural enemies, possible long term damage to ecosystem and human health, and increased production cost [5]. Incorporating BPH resistance genes in rice germplasm into susceptible but otherwise preferred cultivars can be an effective and environmentally friendly approach toward controlling damages caused by BPH [6].

Agronomist have endeavored to identify BPH-resistant germplasm and develop BPH-resistant rice cultivars beginning in the 1960s [7]. At least 30 BPH resistance genes and quantitative trait locis (QTLs) had previously been recognized and incorporated to many rice cultivars [8, 9]. Such approach has been found to be helpful against BPH and led to an improved defense through the incorporation of QTLs. However, it has been quite hard to identify exact roles played by QTLs in the resistance mechanisms against BPH owing to the genomic complexity of the rice cultivars. This has hindered subsequent development of BPH resistant cultivars for specific environments [10]. Analysis of global changes in genes and proteins expression is an approach to learn about the molecular responses happening rice cultivars during BPH stress. It also helps in elucidating various genes and proteins interacting during the defense behavior against BPH, which can be targeted for use in breeding BPH resistant rice [11].

Previous studies based on various transcriptomic and proteomic analyses have revealed that BPH infestation induces complex biological changes affecting the expression of multiple gene and protein regulations in rice. These genetic changes are linked to variations in signaling pathways, wound-responses, and oxidative stress [12]. For instance, during BPH stress condition genes responsible for the production of reactive oxygen species (ROS), stress responses and protein degradation are up-regulated in susceptible rice plants, while those linked to photosynthesis are down-regulated [13].

Recently, a cDNA microarray investigation demonstrated that 1467 differential probe sets may be linked with constitutive resistance [14]. The leaf sheaths of both BPH-sensitive and resistant rice cultivars were found to have over 30 metabolites such as sugars, amino acids, choline metabolites, and organic acids after BPH-induced stress [14]. Advances in transcriptomics and proteomics tools provides unique capability to distinguish plant response to BPH stress and suggests its important role in developing BPH resistant rice [15]. One recent study used a proteomics strategy for the investigation of response given by wild type IR64 and near-isogenic rice mutants with loss and gain of resistance during BPH invasion. It led to the identification of 65 proteins that were remarkably changed during BPH invasion in wild type IR64 [10].

Wild rice species are often resistant to diseases and insect pests but lack desirable agronomic traits, such as plant architecture, grain quality and high yield. Introducing resistance genes from wild species to susceptible rice cultivars can be an important approach for the development of BPH-resistant cultivars [16]. In Yunnan province, China, an important wild species (indigenous) of the genus Oryza - *Oryza officinalis* Wall exWatt (CC, 2n = 2x = 24) is found, which is considered to be a reservoir of several valuable genes for rice breeding, for e.g. resistance to blast, BPH, bacterial blight (BB) and white backed planthopper (WBPH) [17]. A number of resistance genes have been introduced into cultivars through interspecific hybridization and backcrossing between *O. officinalis* and *O. sativa*. Some cultivars have been released for commercial cultivation [18].

In attempt to gain insight into the molecular mechanisms of rice resistance against BPH, in this study, a F1 hybrid rice line (HR) and its highly BPH-resistant maternal *Oryza officinalis* Wall ex Watt line (PR) [19] and BPH-susceptible paternal *Oryza sativa* line Yangdao 6 Hao (PS), were assessed for rice plant responses to BPH attack at the molecular level. This information is useful for understanding the biological basis of BPH resistance and for identification of new BPH resistance-related genes that could be exploited for rice breeding.

## Results

### Rice phenotype during BPH infestation

Following infestation, BPH causes wilting of seedlings, leading to hopper burn symptoms first on susceptible rice line PS,follow by HR and PR (two BPH-resistant lines) (Fig.1 B). Apparent damage to leaves was lowest for PR, intermediate for HR, and highest for PS. Differences in phenotype between susceptible (PS_B) and resistant (PR_B and HR_B) rice lines were quite obvious, consistent with physiological phenotypic results of different resistant rice cultivars after being infected with BPH [20].

**Fig. 1:** Occurrence and symptom of different rice genotypes inoculated by brown rice planthopper. **a** Damage of brown rice planthopper in rice field and typical symptom in dictated at the right corner. **b** Phenotypes of rice genotypes inoculated by brown rice planthopper. Hybrid generations BPH was inoculate with (HR_B) and without (HR) brown rice planthopper; Different lines of hybridization generations BPH, *O. officinalis*, and *O. sativa* were inoculated with brown rice planthopper (HR_B, PR_B, PS_B) while treated without pest as mocks (HR, PR, PS), respectively

### Differentially expressed proteins (DEPs) among three cultivars after inoculations with BPH

Using iTRAQ analysis a total of 4907 proteins were identified from these three cultivars (Additional file 1: Table S1). Between PR and PS, 462 differentially expressed proteins (DEPs) were identified, of which 232 increased and 230 decreased in resistant PR as compared to susceptible PS. Of the 518 DEPs identified between HR and PS, 281 increased and 237 decreased in HR relative to PS. These results indicate wide differences of protein expression in seedlings of these rice cultivars. Inoculation by BPH resulted in significant changes in protein expression in all three rice cultivars: 414 DEPs were detected in PR, of which expression levels of 200 were up-regulated and the remaining 214 down-regulated after inoculation (Additional file 2: Table S2); 423 DEPs were detected in PS, with 248 being up-regulated after inoculation (Additional file 3: Table S3); 190 of 470 DEPs in HR were up-regulated after inoculation (Additional file 4: Table S4) (Fig. 2).

**Fig. 2:** The number of differentially expressed proteins in the three cultivars. The x-axis indicates the comparisons between each two samples. The left y-axis shows the number of differentially expressed proteins

Inoculating with BPH resulted in 1084 identified DEPs (328 + 59 + 21 + 62 + 60 + 280 + 274) among three rice cultivars in response to BPH infection, as shown in the Venn diagram (Fig. 3a). The 21 DEPs shared by HR_B vs. HR, PS_B vs. PS and PR_B vs. PR (Additional file 5: Table S5; Table 1) may confer potential broad-spectrum resistance to BPH [21]. There is a possibility that the 59 DEPs shared by HR_B vs. HR and PR_B vs. PR. are associated with active resistance to BPH by rice [22]. Because one major objective of this study was to screen for internal genetic protein biomarkers involved in resistance to BPH, we selected proteins that are consistently differentially expressed between background and BPH infected plants. We found 15 DEPs shared by four comparison groups of HR_B vs. HR, PR_B vs. PR, PR vs. PS and HR vs. PS (Fig. 3b, Table 2), of which only one (Heat shock protein HSP20, B0FFN6) was significantly up-regulated in every comparison after BPH infection. These results show differences between resistant and sensitive cultivars and further analyses of these genes may shed light on the resistance mechanism.

**Fig. 3:** Venn diagram of DEPs in resistant and susceptible rice cultivars after inoculation with BPH. **a** Venn diagram of comparisons among HR_B-VS-HR, PS_B-VS-PS and PR_B-VS-PR. **b** Venn diagram of comparisons among HR_B-VS-HR, PS_B-VS-PS, PR_B-VS-PR, PR-VS-PS and HR-VS-PS

**Table 1:** Number of the DEPs shown in Fig. 3

DEPs in the Venn diagram	Function of the DEPs	Number of DEPs in the Venn diagram
Among HR_B-VS-HR, PS_B-VS-PS and PR_B-VS-PR	DEPs related to BPH infection	1084
Share by HR_B-VS-HR, PR_B-VS-PR and PS_B-VS-PS	DEPs related to signal transduction after BPH infestation	21
Share by HR_B-VS-HR and PR_B-VS-PR	DEPs related to BPH resistance	59
Share by HR_B-VS-HR, PR_B-VS-PR, PR_VS_PS and HR_VS_PS	DEPs related to marker proteins for rice breeding of BPH resistance	15

**Table 2:** Primers used for quantitative PCR analysis in this study

Uniprot ID	Gene name	Forward primer (5′-3′)	Reverse primer (5′-3′)
Q7EZ84	Os08g0517200	AAATCCGAGCACATGCACAA	CCGACTTCCTGAAGCAAAAC
Q6K832	Os02g0780700	AGCAGGAGCAGGGTGTCAAG	ACATCCTCCGAAGAGTAGCCA
Q6YUV3	Os02g0189100	GATAGTCCGGGCGGTGAATC	AGCATCCAGCTTCTCAAGTACA
Q6AVH9	Os03g0733332	AACCAGGGGTGGGCGAGCTA	ACCGAGCTGTCGCCGAAGCA
Q7XRT6	OSJNBa0042F21.7	AAGCCTTCTGTTGCTCTGCC	TGAAGATGAACCCAACAAAGTG
Q2R1U4	Os11g0592800	GAGGCATACTTGGAGCTTGTG	TTCCGATGAGCATGAGTCTTT
Q6Z7B3	Os02g0115600	GGAAACCCACCATACATCAG	GCACAGATGACTCACGATCA
Q7FAS1	Os04g0623500	CGTCTCCGAGTATGAGCAGC	TGGGCATGGAAATGTTGAAG

To acquire a comprehensive representation of proteomic changes after BHP infestation, all 1084 DEPs were annotated using GO terms and subjected to GO functional analysis. Main biological process categories represented by these DEPs are metabolic processes, stimulus responses, cellular processes and single-organism processes. According to their molecular functional properties, these proteins are mainly classified into catalytic activity, binding, structural molecule activity, electron carrier activity, transporter activity, antioxidant activity and nutrient reservoir activity (Fig. 4). These DEPs were further investigated using the KEGG database and were found to be enriched in biosynthesis of secondary metabolites (10.7%), ribosome (5.0%), carbon metabolism (3.6%), glycosylate and dicarboxylate metabolism (3.2%), porphyrin and chlorophyll metabolism (2.8%), photosynthesis (1.8%), peroxisome (1.8%), carbon fixation in photosynthetic organisms (1.7%), nitrogen metabolism (1.1%), and anthocyanin biosynthesis (0.4%) (Fig. 5).

**Fig. 4:** Gene Ontology (GO) classification of DEPs in rice haulm after BPH infection

**Fig. 5:** Pathway enrichment analysis of DEPs in rice haulm after BPH infection

### Validation using quantitative RT-PCR

For the validation of quantitative results pertaining to correlation between expression patterns of mRNA and their proteins, eight proteins were randomly selected for evaluation of dynamic transcriptional expression profiles using quantitative RT-PCR (Q-PCR) analysis. Table 2 and Fig. 6 show that mRNA expression pattern of the gene encoding Q7FAS1 was similar to the protein expression pattern. Genes Q6AVH9, Q6K832 and Q6Z7B3 in PS_B-VS-PS,HR_B-VS-HR and PR_B-VS-PR groups showed similar expression profiles between mRNA and corresponding protein. On the other hand, genes encoding Q2R1U4,Q6YUV3,Q7XRT6 and Q8H7X8 showed mRNA expression patterns opposite to that of related proteins, which may have resulted from translational or post-translational modifications.

**Fig. 6:** Comparative analysis of protein and mRNA profiles of eight proteins. The x-axis represents comparisons between PS_B and PS, HR_B and HR, PR_B and PR respectively. The left y-axis indicates the relative protein level, whereas the right y-axis pertains to the relative mRNA level. The blue line represents the pattern of protein expression, and the orange line indicates the pattern of mRNA expression

## Discussion

BPH is one of the problematic pests for rice, therefore, it is considered to be a serious threat to large-scale rice production. Breeding resistant cultivars are the most effective and environmentally responsible way for improving crop performance and controlling agricultural pests. In addition, the wild species of the genus *Oryza* possessing ample genetic diversity is still virtually untapped and could, therefore, be used as a key source of BPH resistance [23]. At the present more than 19 BPH-resistance genes have been identified to be assigned with BPH-resistance and assigned to chromosomes of cultivated and wild rice species through QTL mapping [24]. QTL has been used frequently to predict phenotypes for marker-assisted plant breeding. However, the molecular mechanisms that governs main agronomic traits is quite complicated and often requires various stringently controlled processes such as gene regulation, post-translational modifications (PTMs) and protein interactions. The analysis of protein abundance, PTMs, protein-protein interactions, and cellular localization can be facilitated by quantitative proteomics. For the propagation of complex traits that involves protein modifications and its abundance, quantitative protein estimation could be very valuable as markers [25]. In this work, comparative iTRAQ-proteomics analysis was used to identify proteins differentially accumulated in the wild cultivated BPH-resistant rice line PR [19, 26, 27], BPH-susceptible *Oryza sativa* rice line PS, and their BPH-resistant hybrid line HR helped to comprehend the underlying molecular interactions between BPH and rice, as well as inheritable resistance in rice toward BPH. The number of DEPs was considerably elevated as compared to previous studies based on traditional 2D-proteomics [10, 28].

### Proteins participating in early signal transduction after BPH infestation

Signaling pathways of hormones are considered to play crucial roles in the rice defense-signaling network. The defense against BPH in rice and role of plant hormones is quite complex and it varies among genotypes. BPH invasion usually enhances the production of ethylene (Et), salicylic acid (SA), and jasmonic acid (JA) in rice [1]. This study identified 21 DEPs shared by HR_B vs. HR, PS_B vs. PS and PR_B vs. PR comparison groups after BPH inoculation. These DEPs may be involved in early interactions between rice and BPH. It was determined by using the Swissport protein sequence database that these DEPs included 15 proteins of unknown functions, a peroxidase, two Tubulin proteins, two glycosyltransferases and a two-component response regulator protein (ORR22).

The two-component response regulator is related to the two-component system (TCS). The TCS based signal transduction mechanism includes a phosphor relay, which triggers cytokinin signaling. The cytokinin perception results in autophosphorylate of a conserved histidine (H) residue of AHK proteins [29]. Cytokinins are *N*^*6*^-substituted adenine derivatives that were discovered based on their ability to promote cell division in cultured cells. Much progress has been made in understanding cytokinin as an infection signal that activates defense reactions through synergistic action with salicylic acid (SA). Li et al. found that SA content increased significantly after BPH infestation in rice, and that SA plays an crucial role during the rice resistance response against BPH [7]. In this study, the two-component response regulator (ORR22) was markedly up-regulated after infection by BPH, by a factor of 2.61, 9.86 and 1.64 in H, M, and W, respectively, suggesting that ORR22 may play a critical role in resistance to BPH.

### Proteins involved in inheritable resistance of rice against BPH

The identification of proteins involved during parasite attacks and their interactions is necessary in order to understand the basic mechanism of plant resistance. Usually, pathogen-associated proteins have a direct relation to the plant defense processes and are stimulated by pathogen/parasite attack. The sustainability of resistance during compatible and incompatible interactions depends on the interplay of these proteins and the way they accumulate or activate plant defense system [30]. To help understand the inheritable resistance of rice against BPH, we identified 59 DEPs that accumulated in two resistant cultivars (HR and PR) after BPH infestation (Additional file 5: Table S5). Analysis of these 59 DEPs by annotation with the Swissprot database showed that six DEPs related to interaction between rice and BPH all were up-regulated in both resistant cultivars. These six DEPs are considered to be related to inheritable resistance against BPH (Fig. 7).

**Fig. 7:** Fold change of proteins involved in rice inheritable resistance against BPH. The x-axis indicates the protein accession number of Uniprot database. The left y-axis shows the fold change of differentially expressed proteins

A complex defense mechanism has been developed in plants that may employ an organized action of several defense pathways against a variety abiotic and biotic stresses. There are various organic compounds involved in plant defense responses such as oxylipin, ethylene, salicylic acid (SA), etc. [31]. Oxylipins are group of compounds generated by the oxidative modification of polyunsaturated fatty acids that acts as plant messengers. Besides various developmental processes oxylipins are also involved in mediating defense responses against abiotic and biotic stress in crop. The biosynthesis of oxylipin gets initiated by the synthesis of fatty acid hydroperoxides through the oxidation of polyunsaturated fatty acids. To define the first committed step, lipases work in coordination with individual lipoxygenases (LOXs) in different oxylipin biosynthesis pathways [32]. Recent studies on LOX of rice indicated that the up-regulation of LOX could be the main node which mediates JA burst, cross-talk between JA and SA, and trade-offs between resistance to pests [31–34]. In the present study, two LOXs (A2XLT7 and B8BMH5) and one lipases (Q6K832) were found up-regulated in HR and PR after BPH infection, consistent with the idea that LOX is involved in herbivore-induced JA biosynthesis (induced by pests) and is crucial in controlling resistance against chewing and phloem-feeding herbivores in rice.

On the other hand, lignans belong to another class of secondary metabolites which are quite diverse yet broadly distributed in plants and exhibit interesting pharmacological activities. The production of lignans critically involves dirigent proteins (DIRs) and eventually plays a major role in the defense of plants against pests [35, 36]. Plant secondary metabolites act mostly as a regulator of pest feeding however in few other cases they may also control specific physiological functions of insects [35]. An earlier study showed that lignans and stilbenoids can cause moulting disturbances [37]. A recent study on lignans showed that it displays juvenile hormone-like activity that prevents pupal and adult morphogenesis, thus keep insects in their immature state [38, 39]. In the present study, two DIRs (A2Y980 and Q2R0I1) were found to be up-regulated in HR and PR after BPH infection. This may indicate that upon BPH infection, increase of the DIR component promoted contents of lignans and its related secondary metabolites, which might be substances that interfere with growth of BPH [40].

A wide array of defense responses against biotic and abiotic stresses have been developed by plant, among them the production of phytoalexins represent its major chemical defense repertoire [41]. Phytocassanes, recently isolated as rice diterpenoid phytoalexins, is the most abundantly accumulated compound at the edges of necrotic lesions, representing that phytoalexins may help prevent consequent fungal spreading from the infected site [42]. Ent-cassa-12,15-diene synthase (OsDTC1) is thought to have an important function in phytocassanes biosynthesis. OsDTC1 was up-regulated in both HR and PS after BPH infection, which may contribute to elevate levels of phytocassanes and promote resistance to BPH.

### Potential marker proteins for breeding BPH resistant rice

Exploiting resistant cultivars is considered to be an effective and environmentally responsible approach for protecting rice crop from BPH [43]. Traditional breeding methods are limited by genetic complexity, low genetic variance of yield components, inefficient selection methods, environmental variability, and strong genotype-environment interactions [44]. Essentially, several omics-based approaches have enhanced our capability to determine target genetic components and metabolic pathways, which control particular traits and therefore enable us to support selection strategies with screening and analysis platforms [45]. In this study, we found 15 DEPs shared by all pairwise of HR_B vs. HR, PR_B vs. PR, PR vs. PS and HR vs. PS, of which only one (Heat shock protein HSP20, B0FFN6) was found to be significantly up-regulated after BPH infection. Due to various stress conditions small Heat Shock Proteins (sHSPs)/HSP20 gets induced and perform important roles in plant defense against biotic and abiotic stresses s [46]. A recent study showed that small HSP20 of rice is significantly affected by RSV infection, which is transferred through the activity of small brown planthopper (SBPH) in a relentless and circulative-propagative manner [47]. We hypothesize that HSP20 may contribute to a physiologically advantageous response BPH infestation, making it a potential target for marker-assisted selection (MAS) that could significantly improve the efficiency of breeding more BPH resistant rice.

## Conclusions

Combining comprehensive proteomic analysis and qRT -PCR analysis indicated that BPH invasion led to complex protein changes in both BPH- resistant and susceptible rice cultivars. Results of this study provide new hints that will aid to understanding the complex molecular and cellular events in BPH infestation and a potentially useful tool for breeding BPH resistant rice. Responses to BPH infestation that are common to both BPH-resistant and susceptible rice plants are highlighted by activation of ORR22, which may play a role in the resistance response against BPH in early signal transduction through sustained promotion of SA. Importantly, there are substantial differences in inheritable resistance against BPH between resistant and susceptible cultivars—the resistant rice shows drastic reactions to BPH infestation with respect to the number of proteins involved and extent of their changes. LOXs, DIRs and OsDTC1 are key enzyme in inheritable resistance against BPH. In addition, we found that HSP20 could be a potential target for BPH-resistance breeding.

## Methods

### Insect culture and plant material

BPH (*Nilaparvata lugens* Stål) populations were maintained on the susceptible cultivar (*Oryza officinalis,* PS) at the Yunnan Academy of Agricultural Sciences (YAAS), Yunnan Province of China. The initial BPH population was collected from paddy lands nearby YAAS. For invasion, a synchronized hopper stage was obtained using gravid females. The paternal line PS (*O. sativa L.* ssp*. Indica*), the maternal line PR (*O. officinalis*), and their hybrid line HR were used in this study. PR and HR show enhanced defense to BPH infestation while PS is susceptible. Experimental plants were grown at 28 ± 2 °C with a photoperiod of 16 h day/8 h night under greenhouse conditions.

### Plant phenotype to BPH infestation

The study consists of 6 treatments, i.e., *O. officinalis* with (PR_B) and without (PR) BPH infection; *O. sativa* with (PS_B) and without (PS) BPH infection; and their hybrid with (HR_B) and without (HR) BPH infection. Plants were grown until booting stage, when BPH were introduced to three infected treatments. Stem tissues were collected 30 days after BPH infestation began. Visually healthy plants were selected for sampling for treatments without BPH infection. For BPH infected treatments, plants with visual signs of heavy infestation were selected for sampling. Three independent replicates were collected for each treatment. Samples were snap-frozen immediately and kept at − 80 °C until processing.

### Protein extraction

For each plant tissue sample, a 1 g subsample was weighed and homogenized by grinding in liquid nitrogen. The powdered sample was moved quickly to a 50 mL pre-cooled test-tube and then 25 mL precooled acetone (− 20 °C) containing 10% (*v*/v) trichloroacetic acid (TCA) and 65 mM dithiothreitol (DTT) was added. After thorough mixing, the homogenate was precipitated for 2 h at − 20 °C and then centrifuged (16,000×g, 4 °C) for 30 min. The supernatant was removed carefully, and the pellet was then washed thrice with 20 mL chilled acetone (− 20 °C). It was left at − 20 °C for 30 min followed by centrifugation (20,000×g, 4 °C) for 30 min. The precipitation was collected and vacuum freeze-dried. A 250 mg sample of the freeze-dried pellets was weighed and placed in an Eppendorf tube (1.5 mL). The pellets were mixed with SDT lysis buffer (4% SDS, 100 mM Tris-HCl, 100 mM DTT, pH 8.0) and then boiled for 5 min. After boiling the mixture was vortex for 30 s and sonicated intermittently on an ice bath, with 5 s sonication followed by 10 s break, for 5 min at 100 W. The mixture was then boiled again for short time (5 min) and then collected by 30 min centrifugation (12,000×g, 20 °C). The supernatant was collected in a fresh Eppendorf tube (1.5 mL) and passed through a 0.22-μm Millipore filter to collected the lysate. Protein concentration in the lysate was estimated using bicinchoninic acid (BCA) protein assay kit (Beyotime Institute of Biotechnology, China). The rest of the lysate was frozen at − 80 °C until use.

### Protein digestion

Protein digestion was conducted using the FASP procedure [48]. In brief, protein concentrates (300 μg) in an ultrafiltration filtrate tube (30 kDa cut-off, Sartorius, Gottingen, Germany) were mixed with 200 μL UA buffer (8 M urea, 150 mM Tris-HCl, pH 8.0) and centrifuged at 14,000 g at 20°Χ for 30 min. The sample was washed twice by adding 200 μL UA and centrifuged at 14,000 g at 20 °C for 30 min. The flow through from the collection tube was discarded, followed by adding 100 μL IAA solution (50 mM IAA in UA buffer) to the filter tube, mixing at 600 rpm in a thermomixer comfort incubator (Eppendorf, Germany) for 1 min, incubating without mixing for 30 min in the dark at room temperature, and centrifugation at 14,000 g for 30 min at 20 °C. Added 100 μL UA to the filter unit and centrifuge at 14,000 g for 20 min, repeated this step twice. Added 100 μL of a dissolution buffer (Applied Biosystems, Foster City, CA, USA) on the filter, centrifuged at 14,000 g for 20 min, repeated twice. The protein suspension in the filtrate tube was subjected to enzyme digestion with 40 μL of trypsin (Promega, Madison, WI, USA) buffer (4 μg trypsin in 40 μL of dissolution buffer) for 16–18 h at 37 °C. Finally, the filter unit was transferred to a new tube and spun at 14,000 g for 30 min. Peptides were collected in the filtrate and concentration of the peptides was measured by optical density with a wavelength of 280 nm (OD280).

### iTRAQ labeling and high-pH reversed-phased chromatography separation

Digested peptides were labeled with iTRAQ reagents (AB SCIEX, Framingham, MA, USA) following procedures recommended by the manufacturer. Briefly, peptides from sample HR_B, HR, PS_B, PS, PR_B and PR were labeled with iTRAQ reagents 115, 116, 117, 118, 119 and 121, respectively. All labeled peptides were pooled together. Labeled and mixed peptides were subjected to High-pH Reversed-Phase (High-pH RP) Fractionation in a 1100 Series HPLC Value System (Agilent) equipped with a Gemini-NX (Phenomemex, 00F-4453-E0) column (4.6 × 150 mm, 3 μm, 110 Å). Peptides were eluted at a flow rate of 0.8 mL/min. Buffer A consisted of 10 mM Ammonium acetate (pH 10.0) and buffer B consisted of 10 mM Ammonium acetate, 90% *v*/v CAN (pH 10.0). Buffer A and B were both filter-sterilized. The following gradient was applied to perform separation: 100% buffer A for 40 min, 0–5% buffer B for 3 min, 5–35% buffer B for 30 min, 35–70% buffer B for 10 min, 70–75% buffer B for 10 min, 75–100% buffer B for 7 min, 100% buffer B for 15 min and finally 100% buffer A for 15 min. The elution process was monitored by measuring absorbance at 214 nm, and fractions were collected every 75 s. Finally, collected fractions (approximately 40) were combined into 15 pools. Each fraction was concentrated via vacuum centrifugation and was reconstituted in 40 μL of 0.1% v/v trifluoroacetic acid. All samples were stored at − 80 °C until further analysis.

### LC − MS/MS analysis

The 1 μg of each High-pH RP fraction peptides were subjected to Easy-nLC 1000 HPLC system coupled to Orbitrap Elite mass spectrometer (Thermo Fisher Scientific, San Jose, CA, USA). Peptides were separated by Thermo Scientific EASY trap column (100 μm × 2 cm, 5 μm, 100 Å, C18) and analytical column (75 μm × 25 cm, 5 μm, 100 Å, C18). Mobile phase flow rate was 150 nL/min, comprised of Buffer A (0.1% formic acid in water) and Buffer B (0.1% formic acid in 100% ACN). Chromatographic 60 min gradient started from buffer A to 35% buffer B for 50 min, followed by 35–90% Buffer B for 6 min and then 90% Buffer B for 4 min. The mass spectrometer was operated in positive ionization mode. The MS1 spectra of each fraction were acquired between a range of 350–2000 *m/z* at the resolution of 60 K. The 16 most abundant signals from each MS1 spectra were subsequently selected for further fragmentation (MS2) analysis. Data-dependent acquisition (DDA) and higher energy collisional dissociation (HCD) were utilized with a resolution of 15,000 in MS2 analysis. The maximum ion injection times and full scan modes were set 50 ms and 150 ms, 10 × 10^− 6^ and 5 × 10^4^ respectively in MS1 and MS2 analysis. The dynamic exclusion duration was 30s.

### Data analysis

Proteome Discoverer 2.1 (Thermo Fisher Scientific) was used to analyze raw data. Mascot 2.1 (Matrix Science) embedded in Proteome Discoverer was used to search raw data against the Uniprot rice database (October 9, 2016; 168,354 sequences). Search parameters were as follows: monoisotopic mass; trypsin as cleavage enzyme; two max missed cleavages; iTRAQ labeling and carbamido methylation of cysteine as fixed modifications; and oxidation of methionine as variable modifications. Peptide mass tolerance of ±20 ppm and fragment mass tolerance of 0.1 Da were used for parent and monoisotopic fragment ions, respectively. Results were filtered based on a false discovery rate of (FDR) ≤0.01. Relative quantitative analyses of proteins were based on ratios of iTRAQ reporter ions from all unique peptides representing each protein. Relative peak intensities of the iTRAQ reporter ions released in each of the MS/MS spectra were used. Final ratios obtained from relative protein quantifications were normalized based on the median average protein quantification ratio. A reported protein ratio represents the median of ratios of unique peptides of that protein. The mass spectrometry proteomics data have been deposited to the ProteomeXchange Consortium via the PRIDE [49] partner repository with the dataset identifier PXD008926.

### Bioinformatics

Statistical and hierarchical clustering analyses were performed using Perseus V1.4.1.3 [48]. *P*-values of < 0.05 by Benjamini-Hochberg FDR in Perseus and proteins differed by more than 150% between two plant groups were further analyzed for functional and biological relevance. These proteins were classified by their gene functions and also by biological pathways using the freely available gene ontology (GO) database provided by the Gene Ontology Consortium (http://geneontology.org/) [50]. The identified protein sequence information was extracted from the UniProt knowledge base and retrieved in FASTA format. The functional information of the homologous proteins was used to annotate targeted proteins. Top 10 blast hits with E-values of less than 1*e*-3 for each of the query proteins were retrieved and loaded into Blast2GO (Version 2.7.2) [51], a high-throughput online tool for gene ontology (GO) analysis, for GO mapping and annotation. Enriched GO terms were identified with Fisher’s Exact Test. Pathways associated with each identified protein were also annotated according to the KEGG pathway (https://www.genome.jp/kegg/pathway.html). For this study, targeted proteins were blast against the KEGG GENES database using KAAS (KEGG automatic Annotation Server) [52]. Enriched KEGG pathways were identified with Fisher’s Exact Test.

### Validation of protein expression by qRT-PCR

TaKaRa RNAiso reagent (TaKaRa Bio, Otsu, Japan) was used to extract total RNA from six rice samples. The purified RNA was reverse-transcribed into cDNA with M-MLV reverse transcriptase (Promega, Madison, WI, USA) and qRT–PCR reaction was performed in 96-well, 25 μL blocks using the CFX96 Real-time System (BioRad, Hercules, CA, USA). Each qRT-PCR was run in triplicate. Actin (GenBank: AY212324) was used as reference gene to normalize the data and 2-^∆∆CT^ (cycle threshold) method was used to calculate relative expression levels [53].

## Additional files

Additional file 1: **Table S1.** List of 4907 identified proteins in BPH infested rice . (XLSX 610 kb)

Additional file 2: **Table S2.** List of 414 differentially expressed proteins in BPH infested *O. officinalis. (XLSX 35 kb)*

Additional file 3: **Table S3.** List of 423 differentially expressed proteins in *O. sativa* upon BPH infestation. (XLSX 35 kb)

Additional file 4: **Table S4.** List of 470 differentially expressed proteins in hybrid generations upon BPH infestation. (XLSX 38 kb)

Additional file 5: **Table S5.** List of 59 differentially expressed proteins only in resistant cultivars after BPH infestation. (XLSX 24 kb)

## Abbreviations

BB: Bacterial blight
BCA: Bicinchoninic acid
BPH: Brown planthopper
DEP: Differentially expressed protein
DIRs: Two dirigent proteins
HSP20: Heat shock protein
LOXs: Two lipoxygenases
ORR22: Two-component response regulator protein
OsDTC1: Ent-cassa-12,15-diene synthase
QTLs: Quantitative trait locis
ROS: Reactive oxygen species
WBPH: White backed planthopper
YAAS: Yunnan Academy of Agricultural Sciences
